The article "Block Matching Pyramid Algorithm-Based Analysis on Efficacy of Shexiang Baoxin Pills Guided by Echocardiogram (ECG) on Patients with Angina Pectoris in Coronary Heart Disease" was published in 2021. Journal: J Healthc Eng.

# Block Matching Pyramid Algorithm-Based Analysis on Efficacy of Shexiang Baoxin Pills Guided by Echocardiogram (ECG) on Patients with Angina Pectoris in Coronary Heart Disease

**DOI:** 10.1155/2021/3819900

**Published:** 2021-08-06

**Authors:** Junqing Gao, Xu Wang, Lingyan Li, Hong Zhang, Ruiqing He, Bingyu Han, Zongjun Liu

**Affiliations:** Department of Cardiology, Putuo Hospital, Shanghai University of Traditional Chinese Medicine, Putuo District, Shanghai 200062, China

## Abstract

This paper was aimed to explore the application of the block matching pyramid (BMP) algorithm in echocardiographic spot tracking in patients with coronary heart disease (CHD) and angina pectoris, as well as the effect of Shexiang Baoxin pills (a kind of drug containing musk, which is good for cardiac diseases) on blood lipids, cardiac function, and curative effect. 206 patients with CHD angina pectoris in the hospital from July 2018 to May 2020 were selected as the research subjects and were enrolled into the control (Ctrl) group (conventional treatment, *n* = 103) and the observation group (the Shexiang Baoxin pill was given on the basis of conventional treatment, *n* = 103) in random. Then, the patients' echocardiograms were obtained, and the BMP algorithm was used to track the echocardiograms. At 12 months after treatment, the total cholesterol (TC), triglycerides (TG), low-density lipoprotein cholesterol (LDL-C), and high-density lipoprotein cholesterol (HDL-C) were compared. Besides, the differences between left ventricular end-systolic volume (LVESV), left ventricular end-systolic diameter (LVESD), left ventricular end-diastolic volume (LVEDV), left ventricular end-diastolic dimension (LVEDD), cardiac index (CI), cardiac output (CO), and LVEF were observed. Finally, the efficacy of angina pectoris and electrocardiogram was calculated. It was found that the BMP algorithm can track the echocardiograms and display the movement and displacement of the patients' left ventricle. After treatment, in contrast with the Ctrl, the levels of TC, TG, and LDL-C in the observation group were obviously lower (*P* < 0.05); the LVESV, LVEDV, and LVEF were obviously lower (*P* < 0.05), the LVESD, LVEDD, CO, and CI were obviously higher (*P* < 0.05), the total score of angina after treatment was obviously lower (*P* < 0.05), and the total effective rates of angina pectoris and echocardiogram were obviously higher (*P* < 0.05). In conclusion, echocardiographic spot tracking can realize the diagnosis of patients with CHD angina pectoris, and Shexiang Baoxin pill can regulate the blood lipid level and improve the echocardiographic indicators and the clinical efficacy is obvious.

The article "Block Matching Pyramid Algorithm-Based Analysis on Efficacy of Shexiang Baoxin Pills Guided by Echocardiogram (ECG) on Patients with Angina Pectoris in Coronary Heart Disease" was published in 2021. Journal: J Healthc Eng.

## 1. Introduction

In recent years, the incidence and mortality of CHD in China have shown an upward trend year by year, which has seriously threatened people's lives and health. At present, the methods commonly used in clinical treatment of CHD are percutaneous coronary intervention or coronary artery bypass surgery. Surgical treatment can realize the recanalization of the occluded blood vessels, improve the symptoms, and reduce cardiovascular events such as myocardial infarction [1, 2]. The occurrence of CHD angina is correlated with the increase of blood lipid levels and vascular endothelial injury [3]. Therefore, the clinical treatment of CHD not only needs to relieve the symptoms of patients with angina but also needs to control blood lipids and other risk factors for cardiovascular diseases. Traditional Chinese medicine (TCM) has a long history of treating CHD angina pectoris, and studies have confirmed that TCM is better than Western medicine in treating CHD angina. Shexiang Baoxin pill is a TCM preparation, which is developed for clinical treatment of cardiovascular diseases such as CHD [4]. Studies have proved that Shexiang Baoxin pills can improve patients' ECG performance and reduce the incidence of cardiovascular events [5].

Cardiac ultrasound imaging technology is also often used in clinical disease diagnosis and treatment effect evaluation, and the new type of echocardiogram technology can be used for the evaluation of myocardial strain. In addition, it can also measure myocardial deformation [6]. The traditional echocardiographic parameters based on volume measurement are not very sensitive to the early changes of myocardial function, but the spot tracking detection of echocardiogram can realize the assessment of ventricular function in patients with early myocardial diseases [7, 8]. Moinfar et al. used 2-d speckle to track echocardiography. It was found that the left atrial fluid storage and catheter capacity decreased in patients with type 2 diabetes complicated with urinary protein coronary disease [9]. However, there are relatively few studies on echocardiogram in patients with CHD angina.

Therefore, in this study, CHD angina pectoris patients were taken as the research subjects. Then, the patients' echocardiograms were obtained, and the changes of the ventricular function were explored through spot tracking. Subsequently, Shexiang Baoxin pills were given to compare the differences in the blood lipid levels, echocardiographic parameters, and treatment efficiency of different methods. The results provided a reference for improving the clinical treatment of patients with CHD angina.

## 2. Methods and Materials

### 2.1. Research Subjects

206 patients with CHD angina in the hospital from July 2018 to May 2020 were taken as the research subjects. The diagnosis of CHD angina meets the requirements stipulated by WHO. Inclusion criteria: patients must be over 20 years old; patients who clinically demonstrated myocardial ischemia and hypoxia for more than 30 days; and patients who have had acute myocardial infarction for more than 6 months, who have undergone percutaneous coronary intervention or coronary artery bypass surgery, or whose imaging revealed that at least one main branch had a stenosis of more than 50%. At least one of the above events occurred. Exclusion criteria: patients with myocardial infarction or revascularization therapy in the past 6 months; patients with severe respiratory disease; patients with severe other organ dysfunction; patients with serious diseases such as malignant tumors; pregnant women; and patients with severe mental illness. 206 patients with CHD angina were enrolled into the observation group and Ctrl, with 103 in each. Patients in the Ctrl were given conventional treatments, and patients in the other group were given 2 capsules/time and 3 times/d Shexiang Baoxin pills based on the above treatment. This trial had got permission from the ethics committee of the hospital, and the subjects or their families had signed informed consents.

The article "Block Matching Pyramid Algorithm-Based Analysis on Efficacy of Shexiang Baoxin Pills Guided by Echocardiogram (ECG) on Patients with Angina Pectoris in Coronary Heart Disease" was published in 2021. Journal: J Healthc Eng.

### 2.2. Collection of Echocardiograms

The color Doppler ultrasound diagnostic apparatus was adopted to collect the patients' echocardiograms, and the frequency of the S4 probe was set to 2∼4 MHz. During the examination, the probe was needed to be placed between the 3rd and 4th ribs on the left side of sternum to obtain the 4 chambers of the heart. Then, the dimensions of the heart chamber, the thickness of the ventricular wall, the thickness of the left atrium, and contraction and relaxation ability of the left ventricle were observed.

### 2.3. Echocardiogram Spot Tracking Based on Block Matching Algorithm

BMP combines image pyramid and block matching algorithm, which can measure the similarity of image spot position. At the same time, through the sampling of image blocks, there is only a small amount of calculation [10]. The process of BMP algorithm is shown in Figure 1. After the spots to be tracked in the echocardiogram were calibrated, block matching and pyramid models were needed to be built. Then, the SAD value at the current time was calculated, and the similarity of all pixels in the view field was calculated. The comparison ends until all pixels were compared.

In Figure 1, when the BMP algorithm was adopted, the calculation equation of the sum of absolute differences (SAD) value was as follows:

(1) $$\begin{array}{c} {\text{SAD}}_{m}\left(x,y\right)=\sum_{i=1}^{2^{m}}\sum_{j=1}^{2^{m}}\left|x^{m}\left(i,j\right)-y^{m}\left(i,j\right)\right|, \end{array}$$

in which *x*^*m*^(*i*, *j*) represents the value of the pixel at point (*i*, *j*) in the *m*th layer of the pyramid.

The article "Block Matching Pyramid Algorithm-Based Analysis on Efficacy of Shexiang Baoxin Pills Guided by Echocardiogram (ECG) on Patients with Angina Pectoris in Coronary Heart Disease" was published in 2021. Journal: J Healthc Eng.

After the above equation was unfolded and Minkowski's inequality was used, the following equation was obtained:

(2) $$\begin{array}{c} {\text{SAD}}_{m}\left(i,j\right)\geq {\text{SAD}}_{m-1}\left(i,j\right)\geq {\text{SAD}}_{m-2}\left(i,j\right)\geq \cdots \geq \text{SAD}\left(i,j\right). \end{array}$$

### 2.4. Observation Indicators

Blood biochemical indicators and renal function were tested before treatment and 3 months and 12 months after treatment. The patient was in the left decubitus position, and LVESV, LVESD, LVEDV, and LVEDD were collected before and 12 months after treatment. After the collection, the patients' CI, CO, and LVEF were calculated.

### 2.5. Efficacy Criteria

Criteria for determining the effect of angina pectoris: obviously effective (decrease in total angina pectoris points by at least 60%), effective (decrease in total angina pectoris points by at least 30%), ineffective (decrease in total angina pectoris points by less than 30%), and worsening of disease (no decrease in total angina pectoris points).

Criteria for determining the effect of echocardiogram treatment: obviously effective (the echocardiograms returned to the normal range), effective (ST segment was reduced, and after treatment, it rose above 0.05 mV, but did not reach the normal level, or the *T* wave changed from a flat state to an upright state), ineffective (the ECG had no significant changes compared to before treatment), and worsening of disease (the ST segment was reduced by more than 0.05 mV after treatment; the *T* wave state was completely changed, and ectopic heart rate occurred).

### 2.6. Statistics and Analysis

The data were processed by SPSS 20.0. Mean ± standard deviation ($\bar{x}\pm s$) was how measurement data were expressed, and comparison between groups was realized through independent sample t-test. Count data were expressed as frequency or percentage, and the *χ*^2^ test was used to compare differences between groups. When *P* < 0.05, the difference was considered to be statistically significant.

## 3. Results

### 3.1. General Information Comparison

Before treatment, the differences were compared in baseline data, biochemical indicators, and cardiac function indicators. From Table 1, it was evident that there was no obvious difference in baseline data, biochemical indexes, and cardiac function indexes (*P* > 0.05).

### 3.2. Evaluation of Echocardiographic Speckle Tracking Algorithm

First, the difference between the accuracy and time was compared when the global search method or the logarithmic search method was adopted to analyze the pixel points in the motion vector search window in the BMP algorithm (Figure 2). It was evident from Figure 2(a) that the change of the size of search window had a small effect on the search accuracy of the global search algorithm. As the size of search window increased, the accuracy of the logarithmic search method gradually decreased. However, the accuracy rate of the two algorithms was always higher than 90%. It was evident from Figure 2(b) that as the size of search window increased, the running time of the two algorithms gradually increased, but that of the logarithmic search method was always lower than that of the global search method.

The article "Block Matching Pyramid Algorithm-Based Analysis on Efficacy of Shexiang Baoxin Pills Guided by Echocardiogram (ECG) on Patients with Angina Pectoris in Coronary Heart Disease" was published in 2021. Journal: J Healthc Eng.

The heartbeat sequence was selected; each sequence contained 250 frames of heartbeat images and multiple heart motion cycles. It was evident from Figure 3(a) that the red smooth closed contour was the segmentation line of the ventricle and atrium, and the yellow dots around were the marked spots. By tracking these spots, the direction of heart movement was finally obtained (Figure 3(b)). It was evident that the maximum displacement of the heart was about 15 pixels, which was about 13.8 mm.

### 3.3. The Effect of Shexiang Baoxin Pill on Biochemical Indexes

The changes were compared in the levels of biochemical indexes 3 months and 12 months after treatment (Figure 4). It was evident that the levels of biochemical indexes of all patients decreased 12 months after treatment in contrast with those 3 months after treatment. In contrast with Ctrl, at 3 months after treatment, the levels of TC and LDL-C in the observation group were obviously lower (*P* < 0.05); at 12 months after treatment, the levels of TC, TG, and LDL-C were obviously lower (*P* < 0.05). Although the difference in TG levels 3 months after treatment and HDL-C levels 3 months and 12 months after treatment was not obvious (*P* > 0.05), it was observed that those in the observation group were still lower than Ctrl.

### 3.4. The Effect of Shexiang Baoxin Pill on Cardiac Function

The differences were compared in LVESV, LVEDV, LVESD, and LVEDD 12 months after treatment (Figure 5). It was evident that in contrast with Ctrl, the levels of LVESV and LVEDV of the observation group after treatment were obviously lower (*P* < 0.05); the LVESD and LVEDD were obviously higher after treatment (*P* < 0.05) .

The differences were compared in LVEF, CO, and CI 12 months after treatment (Figure 6). In contrast with Ctrl, in Figure 6(a), the LVEF of the observation group after treatment was obviously lower (*P* < 0.05); in Figure 6(b), the CO was obviously higher after treatment (*P* < 0.05); in Figure 6(c), the CI after treatment was obviously higher (*P* < 0.05).

The article "Block Matching Pyramid Algorithm-Based Analysis on Efficacy of Shexiang Baoxin Pills Guided by Echocardiogram (ECG) on Patients with Angina Pectoris in Coronary Heart Disease" was published in 2021. Journal: J Healthc Eng.

### 3.5. Therapeutic Effect Analysis of Shexiang Baoxin Pills

The difference was compared between the total scores of patients with angina before treatment (0 month) and 12 months after treatment (Figure 7). There was no obvious difference in the total score of angina before treatment (*P* > 0.05). After treatment, that in the observation group was obviously lower than Ctrl (*P* < 0.05).

After 12 months of treatment, the difference was compared in the efficacy of angina pectoris and echocardiogram (Table 2). There was no case with aggravated angina pectoris and echocardiogram efficacy in both groups, while the total effective rate of angina pectoris efficacy and echocardiogram efficacy in the observation group was obviously higher than Ctrl (*P* < 0.05).

## 4. Discussion

The occurrence and development of CHD angina are closely related to the ischemia and hypoxia of myocardial cells [11]. At present, many studies have proved that hyperlipidemia is an important factor, leading to a variety of cardiovascular and cerebrovascular diseases [12]. Therefore, in the study, the effect of Shexiang Baoxin pills on the levels of TC, TG, LDL-C, and HDL-C in patients with CHD angina pectoris was explored. It was revealed that at 3 months and 12 months after treatment, the levels of the abovementioned indexes were obviously lower than Ctrl. It was basically in line with the research results of Tian et al. [13], suggesting that Shexiang Baoxin pills can reduce the blood lipid levels in patients with CHD angina pectoris, thereby slowing down the process of coronary atherosclerosis.

Cardiac imaging technology has been widely used in disease prevention, diagnosis, and treatment. Among them, echocardiogram imaging technology has small side effects and is economical. Therefore, it is one of the imaging technologies commonly used in the diagnosis of heart diseases [14, 15]. The echocardiogram spot tracking can realize the assessment of cardiac strain in severe cardiac patients [16]. Therefore, the image pyramid and block matching method were combined to track the echocardiogram of CHD angina pectoris patients in the study. Clinically, the computational complexity of the block matching algorithm makes it difficult to meet the needs of timeliness. Therefore, first, the impact of global search [17] and logarithmic search [18] on the efficiency of the algorithm was analyzed. It was found the tracking accuracy of the two search methods was both higher than 93%. Although the logarithmic search method reduces the tracking accuracy due to the increase of the search window, the tracking time is always lower than that of the global search method. Therefore, the parameters can be adjusted in clinical application to improve tracking effect. When the echocardiograms of patients with CHD angina pectoris were tracked subsequently, it was found that the displacement of the patients' left ventricle could be clearly tracked through the calibrated spots. What's more, the patients' heart motion trajectory showed a certain periodicity, which was in line with the clinical cardiac motion state. However, after tracking, it was found that the maximum displacement of the heart was 15 pixels, about 13.8 mm. Besides, the heart beat was too strong, indicating that the heart function was abnormal. It was in line with the actual situation of CHD angina patients [19].

The article "Block Matching Pyramid Algorithm-Based Analysis on Efficacy of Shexiang Baoxin Pills Guided by Echocardiogram (ECG) on Patients with Angina Pectoris in Coronary Heart Disease" was published in 2021. Journal: J Healthc Eng.

Subsequently, the effect of Shexiang Baoxin pill on the heart function was studied. It was found that the patients in observation group had obviously lower LVESV, LVEDV, and LVEF than the Ctrl (*P* < 0.05), and LVESD, LVEDD, CO, and CI were obviously higher (*P* < 0.05). LVESV, LVEDV, LVEF, LVESD, LVEDD, CO, and CI indicators are important indicators used to evaluate the volume, shape, function, and structure of the heart [20]. It was found that Shexiang Baoxin pills could reduce the left ventricular volume, increase the left ventricular inner diameter, and improve the heart function by increasing cardiac output and enhancing cardiac systolic function. It was in line with the research results of Tian et al. and Zhang et al. [13, 21]. Finally, the difference between the total effective rates of and echocardiogram in two groups was evaluated. It was found that the total effective rates of angina pectoris and echocardiogram in observation were 96.1% and 93.2%, respectively, both of which were obviously higher than Ctrl (*P* < 0.05). It was in line with the results of Chen et al. [22], indicating that the clinical treatment of Shexiang Baoxin pills can obviously improve the symptoms of angina pectoris and enhance the cardiac function of patients, which was consistent with the results of the previous echocardiographic evaluation.

## 5. Conclusion

In the study, the application of the BMP algorithm in echocardiographic spot tracking of patients with CHD angina pectoris, as well as the effect of Shexiang Baoxin pills on blood lipid levels, cardiac function, and treatment efficiency, was explored. It was found that echocardiographic speckle tracking can detect the abnormal displacement of the left ventricle, and giving Shexiang Baoxin pills on the basis of conventional treatment can improve the patients' echocardiographic indicators and increase the total effective rate of treatment. However, only the BMP algorithm is used to realize the echocardiographic speckle tracking. The follow-up studies need to compare and analyze the differences in the results of echocardiographic speckle tracking before and after treatment. In short, the results can provide a theoretical basis for improving the clinical treatment of patients with CHD angina and the quality of life of patients.

The article "Block Matching Pyramid Algorithm-Based Analysis on Efficacy of Shexiang Baoxin Pills Guided by Echocardiogram (ECG) on Patients with Angina Pectoris in Coronary Heart Disease" was published in 2021. Journal: J Healthc Eng.

## Figures and Tables

**Figure 1:** The spots marking process of echocardiograms based on BMP algorithm.

**Figure 2:** Performance comparison of global search method and logarithmic search method. (a) The accuracy rate; (b) the running time.

**Figure 3:** Results of echocardiographic spot tracking. (a) The calibration of echocardiographic spots; (b) the displacement of echocardiographic spots.

**Figure 4:** Comparison of blood lipid indexes after treatment. ^*∗*^ indicates that the difference between groups was obvious, *P* < 0.05 (with the same meaning in Figures 5–7).

**Figure 5:** Comparison of differences in cardiac function indexes after treatment.

**Figure 6:** Comparisons of differences in (a) LVEF, (b) CO, and (c) CI after treatment.

**Figure 7:** Comparison of total scores of angina pectoris.

**Table 1:** Comparison of general information.

Baseline data	Ctrl (*n* = 103)	Observation group (*n* = 103)	*t*/χ^2^	*P* value
Male (case/%)	66 (64.1)	63 (61.2)	1.232	0.153
Age (year)	62.33 ± 8.47	63.28 ± 9.77	0.785	0.229
Course of disease (year)	2.62 ± 1.35	2.53 ± 1.72	0.633	0.314
BMI (kg/m^2^)	22.17 ± 5.43	21.80 ± 4.62	0.791	0.221
TC (mmol/L)	6.52 ± 0.82	6.54 ± 0.67	0.626	0.335
TG (mmol/L)	2.24 ± 0.53	2.35 ± 0.74	0.729	0.304
LDL-C (mmol/L)	4.11 ± 0.58	4.09 ± 0.52	1.223	0.170
HDL-C (mmol/L)	1.35 ± 0.42	1.33 ± 0.21	1.121	0.197
LVESV (mL)	58.92 ± 6.57	58.17 ± 5.93	0.789	0.237
LVESD (mm)	45.83 ± 3.62	44.23 ± 4.11	0.826	0.219
LVEDV (mL)	111.93 ± 10.37	112.76 ± 10.83	0.627	0.335
LVEDD (mm)	66.85 ± 7.68	67.42 ± 8.08	1.109	0.203
CO (L/min)	6.10 ± 1.30	6.00 ± 0.70	1.203	0.188
CI (L/min·m^2^)	4.00 ± 0.20	4.30 ± 0.30	0.668	0.326
LVEF (%)	40.33 ± 4.35	41.63 ± 4.78	0.718	0.315

**Table 2:** Comparison of efficacy between angina pectoris and echocardiogram.

Grade	Angina pectoris efficacy				Echocardiogram efficacy			
	Ctrl (*n* = 103)	Observation group (*n* = 103)	χ^2^	*P* value	Ctrl (*n* = 103)	Observation group (*n* = 103)	χ^2^	*P* value
Obviously effective	41 (39.8)	45 (43.7)	—	—	34 (33.0)	41 (39.8)	—	—
Effective	52 (50.5)	54 (52.4)	—	—	52 (50.5)	55 (53.4)	—	—
Ineffective	10 (9.7)	4 (3.9)	—	—	17 (16.5)	7 (6.8)	—	—
Aggravated	0 (0.0)	0 (0.0)	—	—	0 (0.0)	0 (0.0)	—	—
Effective rate (%)	90.3	96.1	8.325	0.027	83.5	93.2	11.231	0.004

The article "Block Matching Pyramid Algorithm-Based Analysis on Efficacy of Shexiang Baoxin Pills Guided by Echocardiogram (ECG) on Patients with Angina Pectoris in Coronary Heart Disease" was published in 2021. Journal: J Healthc Eng.

## Data Availability

The data used to support the findings of this study are available from the corresponding author upon request.
